# Clothing Design Style Recommendation Using Decision Tree Algorithm Combined with Deep Learning

**DOI:** 10.1155/2022/5745457

**Published:** 2022-08-10

**Authors:** Baojuan Yang

**Affiliations:** Fashion Design Department, Art and Design School, Changchun Humanities and Sciences College, Changchun 130117, Jilin, China

## Abstract

Most clothing recommendation methods have problems such as high resource consumption and inconsistent subjectively labeled clothing labels. Based on this, a multilabel classification algorithm based on deep learning (DL) theory is introduced, based on which the clothing style recognition model is constructed. Next, the concept of the decision tree algorithm is given, and the clothing recommendation model is built based on this algorithm. Moreover, the clothing style recognition model based on a multilabel classification algorithm and the clothing recommendation system based on a decision tree algorithm are tested by building simulation experiments and combining neural network technology. Finally, the application of the decision tree algorithm and DL theory in clothing recommendation design is studied through the literature collection method. The research focus is to realize the recognition of clothing through decision tree algorithm and DL method to achieve the intelligent recommendation of clothing style. The results show that: (1) the neural network technology in DL theory can realize efficient recognition and classification of clothing style by automatically extracting image features and combining with a multilabel classification algorithm. (2) The decision tree algorithm can make an initial recommendation according to users' style preferences, then make implicit recommendations through user retrieval, browsing, and other operations, and make dynamic clothing style recommendations to users. (3) When the neural network based on a multilabel classification algorithm is trained, the precision, recall rate, and F1 values are 0.73, 0.43, and 0.55, respectively. (4) After using the clothing recommendation system based on the decision tree algorithm, the subjects' average satisfaction is 86.25%, indicating that this system can give users a better clothing recommendation experience. This exploration aims to provide a crucial reference for further improving the quality of clothing recommendation services. It has important theoretical significance and practical value for the development of artificial intelligence in the field of fashion design, and is expected to provide a reference for the development of bionics.

## 1. Introduction

Nowadays, with the increasing economic level, people are no longer only satisfied with the clothing requirements for warmth preservation but pursue more clothing styles to dress themselves [1]. However, there is no clear definition and classification standard of clothing style, resulting in differences in the classification of clothing style by different researchers [2]. At present, there are two common classifications of clothing styles. One is to divide clothing into neutral, avant-garde, leisure, sports, classic, elegant, light, and national styles from the perspective of commercial clothing brands. The other is to further subdivide the fashion style from the fashion design perspective. Clothing styles are divided into 18 categories according to cultural and geographical factors, such as Korean version, hip-hop, and street [3]. There are also some other classification methods, such as classifying clothing styles into Gothic, classical, romantic, Baroque, and other styles [4]. According to independent designer brands in different regions, clothing can also be divided into young playful, avant-garde, modern and simple, national retro, elegant, and romantic styles [5]. Thereby, the division of clothing style mainly depends on personal subjective judgment without unified definition standard [6].

Although clothing styles are changeable, people's understanding of the concept of clothing style is not strong [7]. Therefore, the clothing recommendation service of merchants to users is significant [8]. Lots of literature research results show that although great progress has been made in the method of clothing recommendation system, the research on it is not perfect. Jiang et al. proposed that the existing e-commerce websites mainly recommended similar clothing for users through similarity calculation based on users' browsing records, purchase records, and other historical data. Such recommendations are in line with users' preferences, but users rarely buy the same clothes for the second time. Some websites will recommend clothes that hot celebrities or experts think are trendy and popular to users. Although such a recommendation ensures popularity, it does not take into account the uniqueness of everyone. Whether the recommended clothes are suitable for users has certain blindness [9]. Padigela and Suguna pointed out that massive clothing information appeared on the Internet due to the rapid clothing e-commerce development. However, clothing labels are provided by businesses, and the definition of clothing labels is often subjective. Moreover, the classification methods are diverse and complex, so many businesses are difficult to unify, and some labels may be missing or even inconsistent with the images and texts [10]. Mukhametshin et al. held that the clothing recommendation system recommends through keyword searching, which is difficult, affecting the recommendation effect. In recent years, with the proposal of the deep learning (DL) concept, computer vision has been greatly developed. The computer is adopted to analyze and understand image content, simulate human thinking mode, automatically extract image features, and complete image recognition and classification [11]. To sum up, the current clothing classification and recommendation methods are not perfect enough to realize automatic clothing recognition and recommendation. However, DL is currently performing well in visual, speech, and image recognition. The above shows that DL theory can play a crucial role in fashion design recommendations.

To sum up, DL theory is vital for clothing recommendations. Meanwhile, some progress has been made in the clothing recommendation system, but there are still some problems. This exploration introduces multilabel classification and decision tree algorithms based on this. Then, based on these two algorithms, the clothing style recognition model and clothing recommendation model are constructed, respectively. Finally, the experiment is set up to test the two models. The research innovation is to integrate DL and decision tree algorithm, break through traditional clothing image recognition and classification methods, and provide a new method. This exploration aims to provide a theoretical basis for improving the quality of clothing recommendations.

## 2. Materials and Methods

### 2.1. Multilabel Classification Algorithm

The label classification problem can be considered from the algorithm-adaptive method and problem transformation method [12]. The problem transformation method is to transform the multilabel classification problem into multiple single-label classification problems. Finally, the results of multiple single-label classifications are integrated to be the results of multilabel classification to solve the problem of multilabel classification. The algorithm-adaptive method is to transform the existing single-label classification algorithm to realize the function of multilabel classification. The problem transformation method starts from the multilabel classification problem and then converts it to a single-label problem for processing. Thereby, the problem transformation method is to transform the problem form, while the algorithm-adaptation method starts from the single-label problem, and then transforms the problem. However, the principle of the single-label problem remains unchanged, and the problem is processed through the problem transformation [13].

The commonly used evaluation indexes of multilabel image classification are precision, recall rate, and F1 value [14]. Precision refers to the prediction result, which means the probability of actually being a positive sample among all the predicted positive samples. This index measures the proportion of samples with positive prediction in the prediction results, which is a more accurate measure. The higher the precision (closer to 1) is, the better the effect is. The precision represents the prediction accuracy in the positive sample results [15]. Recall rate refers to the probability of being predicted as a positive sample among the actually positive samples. It indicates how many samples of the label in the sample are correctly predicted. It is the ratio of the number of correctly predicted samples in the test set to the total number of samples [16]. Theoretically, the higher the value of precision and recall rate is, the better the classification effect is. However, sometimes, there are extreme situations such as quite high precision but quite low recall rate. F_Measure value is introduced to comprehensively consider the results of the two indexes to avoid the contradiction between them. It is calculated by the weighted harmonic average of precision and recall rate. Therefore, it is a comprehensive calculation method for prediction results and samples [17, 18], expressed as

(1) $$\begin{array}{c} F_{\text{Measure}}=\frac{\left(\alpha^{2}+1\right)\text{Precision}\times \text{Recall}}{\alpha^{2}\left(\text{Precision}+\text{Recall}\right)}. \end{array}$$

When parameter *α* = 1, it is the most common *F*_1_. It reveals that F1 value is the comprehensive result of precision and recall rate. The larger the value is, the better the image annotation performance is [19]. Equations (2)–(4) are the calculation methods of precision, recall rate, and F1 value, respectively. Equation (2) is the calculation method of precision, (3) is the calculation method of recall rate, and (4) is the calculation method of F1 value.

(2) $$\begin{array}{c} \text{Precision}=\frac{1}{\left|N\right|}\sum_{1}^{\left|N\right|}\frac{\sum_{i=1}^{L}y_{i}h_{i}}{\sum_{i=1}^{L}h_{i}},\;\text{Precision}\in \left[0,1\right]. \end{array}$$

*N* represents multilabel samples, |*N*| represents the number of multilabel samples, *L* is the label, and the number of labels is |*L*|. There are |*N*| multiple label samples (*x*_*i*_, *y*_*i*_), *y*=1,2,…, *n*. *x*_*i*_ represents the input data of the sample *i*, *y*_*i*_ is the annotation of the sample *i*, *h*_*i*_ is prediction results for *x*_*i*_. *y*_*i*_ and *h*_*i*_ are the |*L*| dimensional vectors.

(3) $$\begin{array}{c} \text{Recall}=\frac{1}{\left|N\right|}\sum_{1}^{\left|N\right|}\frac{\sum_{i=1}^{\left|L\right|}y_{i}h_{i}}{\sum_{i=1}^{\left|L\right|}h_{i}},\;\text{Recall}\in \left[0,1\right]. \end{array}$$

*F*_1_ is the weighted harmonic average of precision and recall rate:

(4) $$\begin{array}{c} F_{1}=\frac{2\times \text{Precision}\times \text{Recall}}{\text{Precision}+\text{Recall}},\;F_{1}\in \left[0,1\right]. \end{array}$$

However, there is often a certain difference between the label value obtained by the multilabel algorithm and the predicted value. Therefore, the multilabel loss function needs to be introduced [20]. The following is the specific division of the multilabel loss function:

(1) Sigmoid activation function. The nonlinear Sigmoid function is often used in binary classification problems, and its function equation is defined as follows:
  (5) $$\begin{array}{c} S\left(x\right)=\frac{1}{1+e^{-x}}. \end{array}$$
The value range of the output response of the Sigmoid function is compressed to between [0, 1], while 0 corresponds to the “inhibitory state” of biological neurons and 1 corresponds to the “excited state.”
(2) Binary cross-entropy loss function. The Sigmoid activation function is adopted and its output is taken as the input of the binary cross-entropy loss function, which can speed up the network's training. It is set that: there are *N* training samples for an image classification task. *x*_*i*_ is the input feature of the *i*-th sample in the last classification layer of the network. The real mark corresponding to this sample is *y*_*i*_ ∈ {0,1}. *z*_*θ*_(*x*_*i*_ is the prediction result of input characteristic *x*_*i*_. *θ* is the model parameter. Then, the calculation of the binary cross-entropy loss function is
  (6) $$\begin{array}{c} \text{BCE}=-\left[\sum_{i-1}^{N}y_{i}\text{log}z_{\theta }\left(x_{i}\right)+\left(1-y_{i}\right)\text{log}\left(1-z_{\theta }\left(x_{i}\right)\right)\right]. \end{array}$$
Among them, equations (1)–(4) are the indexes to evaluate the model, and (5) and (6) are to calculate the cross-entropy loss. Based on this, the model can be optimized to improve the calculation effect of the model and comprehensively optimize the performance of the model. The calculation of *z*_*θ*_(*x*_*i*_) reads:
  (7) $$\begin{array}{c} z_{\theta }\left(x_{i}\right)=\frac{1}{1+e^{-\theta^{T}x_{i}}}. \end{array}$$
(3) Sigmoid cross-entropy loss function. The average cross-entropy *L* between the predicted value *z*_*θ*_(*x*_*i*_) and the real value *y* is
  (8) $$\begin{array}{c} L=-\frac{1}{N}\left[\sum_{i-1}^{N}y_{i}\text{log}z_{\theta }\left(x_{i}\right)+\left(1-y_{i}\right)\text{log}\left(1-z_{\theta }\left(x_{i}\right)\right)\right.. \end{array}$$

### 2.2. Decision Tree Algorithm

Decision tree learning is a case-based inductive learning algorithm. It infers the classification rules of the form of a decision tree from a group of unordered and irregular cases. It is usually used to form classifiers and prediction models, which can classify, predict, or mine location data [21]. It consists of two steps. The first step is to use the training sample set to establish and refine a decision tree and build a decision tree model. It is a process of acquiring knowledge from data and machine learning. It is usually divided into two stages: tree building and pruning. The second step is to use the established decision tree to classify the new data [22].

Figure 1 is the tree-building process of the decision tree. *S* represents the training sample set, *A* represents the classification sample set, and *N* represents a classification leaf node.

Figure 1 displays that the task of the decision tree pruning phase is to prune the generated decision tree according to certain methods. Pruning is a basic technology to overcome the data noise of the training sample set. When pruning and optimizing the tree, it is necessary to accurately understand the classification feature description and prevent too much noise to achieve a better pruning effect and improve comprehensibility while ensuring accuracy [23, 24]. A decision tree-based classification algorithm is widely used because of its unique advantages.  Figure 2 shows its advantages.

Figure 2 reveals that, first, the structure of the decision tree method is simple, and it does not need to know a lot of background knowledge in the learning process. Second, it has high efficiency and is suitable for the case of a large amount of data in the training sample set. Third, its amount of computation is relatively small. Fourth, it usually does not need the knowledge outside the trained data, and is good at dealing with non-numerical data. Finally, it has high classification accuracy. According to statistics, its utilization rate is as high as 19%.

Among the classification algorithms of decision trees, the early ones are the Concept Learning System (CLS) and Classification and Regression Trees (CART) algorithm [25]. The most influential is the Iterative Dichotomiser 3 (ID3) algorithm. Based on the ID3 algorithm, the C4.5 algorithm is proposed [26]. Several improved algorithms are proposed later to meet the needs of processing large-scale data sets, such as the Supervised Learning In Quest (SLIQ) algorithm and the Scalable Parallelizable Induction of Classification Tree (SPRINT) algorithm [27]. Among the above algorithms, the ID3 algorithm is the representative of the decision tree algorithm, and most decision tree algorithms are improved on its basis. It adopts the “divide and conquer” strategy [28]. When selecting attributes on all levels of nodes in the decision tree, it uses information gain as the selection standard of attributes, so that when testing on each nonleaf node, it can obtain the largest category information about the tested records [29]. The information gain is calculated as follows. *S* is set as a set of *s* data samples. If the class label attribute has *m* different values, *m* different classes *C*_*i*_(*i* = 1,…, *m*) are defined. *S*_*i*_ is set as the number of samples in class *C*_*i*_, and the expected information required for classifying a given sample is

(9) $$\begin{array}{c} I\left(S_{1},S_{2},\ldots ,S_{m}\right)=-\sum_{i=1}^{m}p_{i}lb\left(p_{i}\right), \end{array}$$

where *p*_*i*_ is the probability that any sample belongs to *C*_*i*_. It is set that attribute *A* have *v* different values {*a*_1_, *a*_2_,…, *a*_*y*_}. *S* can be divided into *v* subsets {*S*_1_, *S*_2_,…, *S*_*v*_} by attribute *A*. Among them, the samples in *S*_*j*_ have the same value *a*_*j*_(*j* = 1, 2,…, *v*) on attribute *A*. *S*_*ij*_ is set as the number of samples of class *C*_*i*_ in subset *S*_*j*_, and the entropy or information expectation of the subset divided by *A* is

(10) $$\begin{array}{c} E\left(A\right)=-\sum_{j=1}^{v}\frac{S_{1j},S_{2j},\ldots ,S_{mj}}{S}I\left(S_{1j},S_{2j},\ldots ,S_{mj}\right). \end{array}$$

Equations (9) and (10) are the information gain obtained by branching sample *S* on attribute *A*, which is recorded as *Gain*(*A*) [30].

### 2.3. Design of Clothing Style Recognition Model Based on DL Multilabel Classification

In the field of machine learning, a common kind of work is to use labeled data to train neural networks for classification, regression, or other purposes. This method of training model learning rules is generally called supervised learning. In supervised learning, the quality of labels corresponding to training data is crucial for the learning effect. If the label data used in learning are all wrong, it is impossible to train an effective prediction model. Meanwhile, the neural network used in DL is often complex in structure. In order to obtain good learning results, there are also high requirements for the number of training data with labels, that is, the often mentioned big data or massive data. The core of image classification is to assign a label to an image from a given classification set. In fact, this means that the task is to analyze an input image and return a label that classifies the image. Labels are always from a predefined set of possible categories. There may be *n* categories in the given image to be classified. It is quite a tedious process to manually check and classify the image. Therefore, it is crucial to classify images according to labels through DL technology, which can realize automatic image classification, improve the efficiency of image classification, and optimize the effect of image classification.

The image of the multilabel classification clothing dataset comes from the dataset of the clothing style classification problem. Based on the original clothing style label, the labels of clothing's main color, collar type, looseness, category, and suitable season of clothing are added [31].  Table 1 shows the specific quantity distribution of labels.

Table 1 shows that the total number of labels is 35. The 35 labels are saved as a sequence table file. The label number starts from 0 to 34, and the file is stored in text format.  Figure 3 shows the specific division of labels of clothing images.

Figure 3 reveals that there are multiple types of labels for clothing images, and clothing can be identified through various labels. The accuracy of clothing recognition is improved through the accurate division of labels.  Figure 4 shows the Comma Separate Values (CSV) file format corresponding to the image and label.

Figure 4 suggests that the first column represents the name of the clothing image, and the second column represents the label of the clothing image. All image corresponding labels from the dataset are processed into an array in the one-hot coding format. The array order corresponds to the column order of the clothing image label file. The array shape is (35446, 40), and each line in the array represents the label of an image, corresponding to the content order in the label text. If the label position is 1, it means that the image has the label, and if it is 0, it means that the image does not have the label.

### 2.4. Design of Clothing Recommendation Model Based on Decision Tree Algorithm

According to the characteristics of clothing and users' information data, the decision tree method is adopted for the initial recommendation of clothing style.  Figure 5 is a decision tree.

Figure 5 displays that the decision tree algorithm used has a three-layer tree structure, and the root section of the first layer represents users. The second layer is based on the user's gender. People of different genders have different preferences for clothing styles. For example, female users may like the light style, while male users will not choose the light style. The third layer is based on the user's style preference attributes. Here, six preference attributes are selected: age, collar type, profile, sleeve type, color, and fabric.

First, the eight clothing styles correspond to the letters *T*_1_, *T*_2_, *T*_3_, *T*_4_, *T*_5_, *T*_6_, *T*_7_, and *T*_8,_ respectively.  Figure 6 presents the corresponding relationship.

In Figure 6, based on the eight styles of clothing, the six attributes of clothing style preference can also be transformed into a set. Set A represents age, set B represents collar type, set C represents profile, set *D* represents sleeve type, set *E* represents fabric, and set F represents the color. Then, the A-F style indexes are further refined: *A* = {*a*_1_, *a*_2_, *a*_3_, *a*_4_}, *B* = {*b*_1_, *b*_2_, *b*_3_, *b*_4_, *b*_5_, *b*_6_, *b*_7_}, *C* = {*c*_1_, *c*_2_, *c*_3_, *c*_4_, *c*_5_}, *D* = {*d*_1_, *d*_2_, *d*_3_, *d*_4_, *d*_5_, *d*_6_}, *E* = {*e*_1_, *e*_2_, *e*_3_}, and *F* = {*f*_1_, *f*_2_}. Among them, *a*_i_ represents different age groups, *b*_i_ represents different styles of collars, *c*_i_ represents different types of silhouettes, *d*_i_ represents different styles of sleeves, *e*_i_ represents fabrics of different materials, and *f*_i_ represents different clothing colors.  Figure 7 shows the distribution of specific indexes.

Figure 7 proves that the decision tree algorithm adopted has certain advantages. (1) The decision tree algorithm is easy to understand and the mechanism is simple to explain. (2) The algorithm can be used for small datasets. (3) Its time complexity is small. (4) Compared with other algorithms, the decision tree algorithm can deal with data classification problems. (5) It can handle the problem of multiple outputs. (6) It is insensitive to the missing values. (7) It can process irrelevant feature data. (8) Its efficiency is high. The decision tree only needs to be built once and used repeatedly. The maximum number of calculations for each prediction does not exceed the depth of the decision tree. Therefore, the decision tree algorithm can improve the efficiency of fashion design.

### 2.5. The Influence of Technology on Clothing

Clothing material is a very crucial part of clothing design. The combination of various clothing materials will make the final designed clothing that show different styles and performance effects to meet the diversified needs of consumers [32]. Recently, with the continuous progress of the level of science and technology, many science and technology have been applied in fashion design. In the fashion design process, fashion designers can use high-quality scientific and technological materials to promote the diversification of clothing patterns, colors, and luster to bring new visual effects to users. The scientific and technological materials widely used in the current fashion design process include Lycra fiber, color-changing fiber, and shape memory fiber. The use of modern technology can make clothing present the following characteristics. First, the collocation of clothing decoration develops towards the direction of simplification. Meanwhile, the material and texture of clothing become more and more high quality. Next, the functional services of clothing begin to increase, and the mood of clothing design begins to highlight. Finally, the rapid modern clothing development also puts forward relevant requirements for the use of science and technology. Hence, clothing designers should have advanced design concepts to design high-quality clothing to meet the needs of consumers [33].

The influence of science and technology on fashion design is mainly reflected in two aspects. (1) Personalized needs of consumers. With people's life quality improvement, consumers begin to pursue the fashion and personalization of clothing, so the use of modern technology in clothing design is crucial. If fashion designers want to improve the performance of clothing, enrich the color of fabrics, and improve the texture of clothing, they need to strengthen the use of modern technology. Consumers have higher requirements for modern fashion design with modern science and technology development. Therefore, only through artistic treatment and the innovative design of clothing materials and shapes, can fashion designers meet the personalized needs of different consumers. For fashion designers, the use of scientific and technological materials can help them design fashion products that lead the trend to improve market competitiveness and attract consumers' attention [34]. (2) The determinants of fashion design. The elements of modern fashion design mainly include material use, color matching, and shape design, among which the use of fashion materials is crucial. The choice of clothing materials will diversify the clothing style and give consumers various skin touches. The drape and elasticity of clothing materials will also affect clothing modeling. Hence, if fashion designers want to design high texture and high elasticity clothing products, they should integrate modern science and technology into fashion design to improve clothing performance. For example, in the fashion design process, scientific and technological elastic materials, such as Coolmax fiber and Lycra fiber, can be used. This scientific and technological elastic material belongs to man-made fiber, which can expand clothing tension by 4∼7 times after being applied to fashion design. In addition, it can also give clothing properties such as mildew resistance, hydrolysis resistance, and moth resistance to improve the softness of clothing materials [35].

Meanwhile, this exploration also hopes to contribute to the development of bionics. Bionics is a subject to realize and effectively apply biological functions in engineering. For example, with regard to information reception (sensory function), information transmission (neural function), and automatic control system, the structure and function of this organism have given great inspiration in mechanical design. As an independent discipline, bionics was officially born in September 1960. The first bionics conference was held by the US Air Force Aviation Administration at the air force base in Ohio. The central topic discussed at the meeting was “can the concepts obtained from the analysis of biological systems be applied to the design of artificial information processing systems?” Steele named the emerging science “Bionics,” which in Greek means the science of studying the functions of the life systems. Therefore, this exploration is also a factor in the development of bionics to a certain extent, so it has a certain role in promoting the development of bionics.

## 3. Results and Discussion

### 3.1. Performance of Clothing Style Recognition Algorithm Based on Multilabel Classification

The experimental evaluation indexes of the label clothing classification algorithm are precision, recall rate, and *F*_1_ value. The evaluation index values of each iteration of the neural network based on this algorithm are recorded during the experiment.  Figure 8 shows the results.

Figure 8 suggests that at the beginning of training, the evaluation index values of the network rise sharply, then fluctuate slightly near the highest value and gradually stabilize. When the network achieves the best performance, the precision, recall rate and *F*_1_ values are 0.73, 0.43, and 0.55, respectively. Before the network reaches the best performance and tends to be stable, the starting point of the network is not 0, and the slope of each evaluation index curve is quite large. It shows that the initial performance of the network is better, the convergence speed is faster, and the effect is better. *F*_1_ value of the algorithm is high, indicating the effectiveness of the multilabel clothing classification algorithm.

### 3.2. Test Results of Clothing Recommendation Model Based on Decision Tree Algorithm

Twenty users aged 18–45 are invited to test the clothing recommendation model based on the decision tree algorithm.  Figure 9 shows the feedback results obtained.

Figure 9 reveals that in the 30 recommendation tests of 20 groups, the number of users'satisfaction is generally more than 20, and the maximum number of users' satisfaction can reach 30, indicating that the recommendation results are relatively ideal. Moreover, the average satisfaction of 20 users is 86.25%, which suggests that the overall recommendation effect is good. However, some users' satisfaction is still below 80%. The reason may be that the sample is not perfect enough to fully meet the subjects' needs, thus affecting the satisfaction of the recommendation. Next, it may be that the clothing style attributes have a cross-influence on the clothing style, resulting in the deviation of the overall preference of the subjects for clothing. Finally, it may also be that the subjects' preference for clothing style is low, resulting in fewer styles that meet the recommendation conditions when the system recommends styles, so the recommendation satisfaction is low.

## 4. Conclusion

With the development of the times and the constant changes of people's aesthetics, clothing recommendation service has become an inevitable demand of life. However, there are many problems in traditional clothing recommendations, such as large work demands, easy-to-make mistakes in clothing label labeling, and so on. Therefore, it is particularly important to integrate scientific and technological means into the clothing recommendation system. The research results reveal that: (1) decision tree algorithm and neural network technology in DL theory play an essential role in the optimization of clothing recommendation system; (2) when the neural network based on multilabel classification algorithm is trained, the evaluation indexes of the network tend to be stable gradually, the initial performance of the network is good, and the convergence speed and effect are also significantly improved; (3) when testing the clothing recommendation system based on decision tree algorithm, in the test of user satisfaction times, the number of user satisfaction times in 30 recommendation results is generally more than 20 times and the average value of user satisfaction is more than 85%. It shows that the clothing recommendation system based on a decision tree algorithm has a good effect and can give users a better clothing recommendation experience. The research deficiency is that the experimental samples are not perfect, and the subjects' needs are not well met, which has a certain impact on the experimental results. This exploration aims to provide a theoretical basis for further improving the performance of the clothing design recommendation system.

## Figures and Tables

**Figure 1:** Tree building flowchart of decision tree.

**Figure 2:** Advantages of the decision tree algorithm.

**Figure 3:** Content frame of the clothing image label.

**Figure 4:** Correspondence between image and label file format.

**Figure 5:** Decision tree based on clothing recommendation model.

**Figure 6:** Clothing styles corresponding to different letters.

**Figure 7:** Specific indexes of various attributes in clothing style.

**Figure 8:** Index values of neural network based on multilabel classification algorithm.

**Figure 9:** Test results of clothing recommendation system based on decision tree algorithm: (a) comparison between the number of recommended clothes and the number of clothes satisfied by users; (b) user satisfaction distribution.

**Table 1:** Distribution of the number of clothing labels.

Label name	Basic clothing	Advanced clothing	Season for clothing	Collar type	Looseness	Color
Number of labels	5	7	4	8	3	8

## Data Availability

The datasets used and/or analyzed during the current study are available from the corresponding author on reasonable request.

## References

[1] Ma T. (2021). Research on clothing design based on 5G network and FPGA. *Microprocessors and Microsystems*.

[2] Mu X., Li C. (2021). Research on clothing rental model under sharing economy. *E3S Web of Conferences*.

[3] Chen S. S. (2021). Exploration on the new direction of fashion design from the perspective of youth subculture—doll clothing as example. *Open Access Library Journal*.

[4] Salvadori M., Sbrolli C. (2021). Wall paintings through the ages: the roman period-Republic and early Empire. *Archaeological and Anthropological Sciences*.

[5] Papachristou E., Chrysopoulos A., Bilalis N. (2020). Machine learning for clothing manufacture as a mean to respond quicker and better to the demands of clothing brands: a Greek case study. *International Journal of Advanced Manufacturing Technology*.

[6] Ryding D., Claudia C. E., Vignali G. (2020). Extending the consumer style inventory to define consumer typologies for secondhand clothing consumption in Poland. *European Research Studies Journal XXIII*.

[7] Li Y., He Z., Wang S., Wang Z., Huang W. (2021). Multideep feature fusion algorithm for clothing style recognition. *Wireless Communications and Mobile Computing*.

[8] Mezni H., Benslimane D., Bellatreche L. (2021). Context-aware service recommendation based on knowledge graph embedding. *IEEE Transactions on Knowledge and Data Engineering*.

[9] Jiang S., Zhang Y., Xu H. (2020). Personalized recommendation method of E-commerce based on fusion technology of smart ontology and big data mining. *IOP Conference Series: Materials Science and Engineering*.

[10] Padigela P. K., Suguna R. (2021). Segmentation of E-commerce users based on cart abandonment and product recommendation through collaborative filtering: the moderating effect of exorbitant pricing. *International Journal of System Assurance Engineering and Management*.

[11] Mukhametshin A., Grakhova S., Zakharova I., Belyaeva N., Okisheva K. (2021). Historical insight on provincial merchants of the late 19th century. *E3S Web of Conferences*.

[12] Li S., Xu D., Liu Y., Rui W., Jian Z. (2022). Identification Method of Influencing Factors of Hospital Catering Service Satisfaction Based on Decision Tree Algorithm. *Applied Bionics and Biomechanics*.

[13] Liao Y., Xiong S., Huang Y. (2021). Research on fire inspection robot based on computer vision. *IOP Conference Series: Earth and Environmental Science*.

[14] Tu M., Xu S. (2020). Multi-label text classification algorithm based on semi-supervised learning. *Journal of Physics: Conference Series*.

[15] Yang H., Jiao S. J., Yin F. D. (2020). Multilabel image classification based fresh concrete mix proportion monitoring using improved convolutional neural network. *Sensors*.

[16] Kolisnik B., Hogan I., Zulkernine F. (2021). Condition-CNN: a hierarchical multi-label fashion image classification model. *Expert Systems with Applications*.

[17] Zhou J., Ran F., Li G., Peng J., Kun L., Zheng W. (2022). Classroom Learning Status Assessment Based on Deep Learning. *Mathematical Problems in Engineering*.

[18] Zhao H., Zhou W., Zhu X., Zhu H. (2020). Double attention for multi-label image classification. *IEEE Access*.

[19] Barakaz F. E., Boutkhoum O., Moutaouakkil A. E. (2021). A hybrid naïve Bayes based on similarity measure to optimize the mixed-data classification. *TELKOMNIKA (Telecommunication Computing Electronics and Control)*.

[20] Gong J., Ma H., Teng Z. (2020). Hierarchical graph transformer-based deep learning model for large-scale multi-label text classification. *IEEE Access*.

[21] Liu Q. X., Xia X. (2022). Construction of classification model of academic library websites in jiangsu based on decision tree algorithm and link analysis method. *Open Access Library Journal*.

[22] Qian Z., Liu X., Tao F., Zhou T. (2020). Identification of urban functional areas by coupling satellite images and taxi GPS trajectories. *Remote Sensing*.

[23] Qiu J., Ma L. (2021). Fusion Mode and Style Based on Artificial Intelligence and Clothing Design. *Mathematical Problems in Engineering*.

[24] Mijwil M. M., Abttan R. A. (2021). Utilizing the genetic algorithm to pruning the C4.5 decision tree algorithm. *Asian Journal of Applied Sciences*.

[25] Pandhita S. G., Sutrisna B., Wibowo S. (2020). Decision tree clinical algorithm for screening of mild cognitive impairment in the elderly in primary health care: development, test of accuracy, and time-effectiveness analysis. *Neuroepidemiology*.

[26] Jiang J., Zhu X., Han G., Guizani M., Shu M., Shu L. (2020). A dynamic trust evaluation and update mechanism based on C4.5 decision tree in underwater wireless sensor networks. *IEEE Transactions on Vehicular Technology*.

[27] Zhang J., Xia K., He Z., Shurui F. (2020). Dynamic Multi-Swarm Differential Learning Quantum Bird Swarm Algorithm and its Application in Random Forest Classification Model. *Computational Intelligence and Neuroscience*.

[28] Mao L., Zhang W. (2021). Analysis of entrepreneurship education in colleges and based on improved decision tree algorithm and fuzzy mathematics. *Journal of Intelligent and Fuzzy Systems*.

[29] An Y. B., Zhou H. (2022). Short term effect evaluation model of rural energy construction revitalization based on ID3 decision tree algorithm. *Energy Reports*.

[30] Li Y., Shi F., Hou S., Li J., Li C., Yin G. (2020). Feature pyramid attention model and multi-label focal loss for pedestrian attribute recognition. *IEEE Access*.

[31] Cao C. (2022). Research and application of 3D clothing design based on deep learning. *Advances in Multimedia*.

[32] Pakhomova S. A., Fakhurtdinov R. S., Tsinkolenko O. A., Zolotov B. S. (2020). The influence of carburization technology on performance properties of high-loaded gear wheels. *IOP Conference Series: Materials Science and Engineering*.

[33] Chen J., Yang M., Guo Y., Zhang H. (2021). Innovation ability cultivation of graduate students of computer science and technology under the background of science and education integration. *Advances in Applied Sociology*.

[34] Xiang X. T. (2021). Factors that influence consumers’ behaviors in fashion market. *Open Journal of Business and Management*.

[35] Shindy S., Hariandja E. S. (2021). The influence of brand credibility towards words of mouth of fashion brand. *Journal of Economics, Business, & Accountancy Ventura*.

